# Mangosteen vinegar from Garcinia mangostana: quality improvement and antioxidant properties

**DOI:** 10.1016/j.heliyon.2022.e11943

**Published:** 2022-12-13

**Authors:** Nathamon Suksamran, Visaka Anantawat, Phanphen Wattanaarsakit, Chen Wei, Md. Atiar Rahman, Hideyuki J. Majima, Jitbanjong Tangpong

**Affiliations:** a Department of Food Technology, School of Agricultural Technology, Walailak University, Nakhon Si Thammarat, 80160, Thailand; b Department of Pharmaceutics and Industrial Pharmacy, Faculty of Pharmaceutical Sciences, Chulalongkorn University, Bangkok, 10330, Thailand; c College of Biosystems Engineering and Food Science, Zhejiang University, Hangzhou 310058, PR China; d Department of Biochemistry and Molecular Biology, University of Chittagong, Chittagong, Bangladesh; e School of Allied Health Sciences, Walailak University, Nakhon Si Thammarat, 80160, Thailand; f Research Excellence Center for Innovation and Health Products: RECIHP, Walailak University, Nakhon Si Thammarat, 80160, Thailand

**Keywords:** Mangosteen vinegar, Quality improvement, Antioxidant activity, Phenolic contents, Sensory evaluation

## Abstract

Mangosteen (*Garcinia mangostana* Linn.) fruit is rich in phenolic compounds which function as antioxidants and play a role in anti-inflammation, anti-hyperlipidemia, and anti-diabetic nephropathy. To investigate mangosteen vinegar (MV) by steaming under high pressure, explore the effects of fermentation, antioxidant activity, and sensory evaluation acceptable using the 9 -point Hedonic scale. Steamed mangosteen was processed to produce 3 types of mangosteen vinegar: mangosteen rind vinegar (MRV), mangosteen flesh vinegar (MFV), and mangosteen rind plus flesh vinegar (MRFV). All 3 kinds of mangosteen vinegar were obtaining >4% acetic acid and significantly higher total phenolic content (TPC), total flavonoid content (TFC), and free radical scavenging ABTS+ and DPPH- antioxidant activity than apple cider vinegar (ACV) (*p* < 0. 05). The phenolic compounds analysis of mangosteen vinegar using HPLC were found Gallic acid, Catechin, Epicatechin, Vanillic acid, Trans-ferulic acid, Rutin, Gamma-mongostin, and Alpha-mangostin which showed almost higher than that found in ACV. Therefore, MVs produced from streamed mangosteen have higher antioxidants and were more acceptable using the 9-point Hedonic scale, a significantly higher statistical analysis of sensory evaluation than ACV, especially MFV. Taken together, steamed MVs should be further studied to prove the health benefits as a dietary supplement.

## 1 Introduction

Mangosteen or *Garcinia mangostana* is a tropical fruit belonging to the Clusiaceae family. The fruit was used as traditional herbal medicine for a long time because of the phenolic substance including xanthones, tannin, and pro-anthocyanin [1, 2]. The color intensity of mangosteen fruit is an increase during the ripening period, which is associated with increased xanthones concentration. According to the previous study, higher concentrations of xanthones are available in the peel of purple-black fruit [3]. Xanthone derivatives of *G*. *mangostana* have been reported for neuroprotection against lead-induced acetylcholinesterase (AChE) dysfunction and cognitive impairment in mice [4]. Xanthones remarkably protect against lead-induced chronic kidney disease (CKD) by activating Nrf-2 and modulating NF-kB, MAPK pathways, and improving the tissue architecture [5]. Extract of mangosteen pericarp (rind or peel) has been shown to have various potent pharmacologic properties including antioxidant, antibacterial, antiviral, anti-allergic, anti-proliferative, anti-carcinogenic, and anti-inflammatory properties [6, 7].

According to Food and Agriculture Organization of the United Nations (FAO) reported, the export of this fruit to world markets results in a major economic impact with nearly 400,000 tons produced in Thailand in 2022 [8]. However, the purple-black fruit, a final ripening stage, which is the main problem for mangosteen exporters, and peel is originally a by-product. Mangosteen-derived products such as vinegar or extract are the most popular in the form of beverages, which are sold in the market for health benefits. Previous studies in our laboratory has been the first to report that mangosteen vinegar rind (MVR), a polyphenol-rich natural product from the mangosteen fruit pericarp, prevents a high-fat diet and streptozotocin-induced Type II diabetes nephropathy and apoptosis in albino mice [9]. Vinegar is a liquid that contains 4–20% acetic acid (CH_3_COOH), water, and other substances. Acetic acid was produced through the processing of fermentation using yeast to convert sugar to ethanol, alcoholic fermentation, and followed by acetic acid bacteria such as Acetobacter species which convert ethanol to acetic acid, acetic fermentation, the production of vinegar [10, 11].

Fruit vinegar comes in several flavors, including apple, grape, blackcurrant, raspberry, quince, mango, kaki, berries, and kiwi, and is prepared from a variety of raw materials such as malted barley, balsamic, and rice derived from fruit wine [12]. Traditional fruit vinegar such as pineapple, banana, papaya, mango, longan, and mangosteen vinegar is produced in Thailand. The main component of vinegar in the global market usually is acetic acid, which ranges from 4-8%, and gives a pungent aroma and a sour taste. Acetic acid is mainly found in vinegar, which is obtained by probiotic acetic acid bacteria, *Acetobactor acetate*, and fermentation that bring vinegar beneficial to human intestinal health [13]. The other constituents of vinegar include other organic acids such as citric acid, malic acid, lactic acids, alcohols, vitamins, mineral salts, amino acids, as well as polyphenol compounds with antioxidant properties [14]. Phenolic compounds can reduce free radicals and exert protective effects against oxidative stress and inflammation in the body of consumers delayed aging and a decreased risk of chronic disease [15].

Vinegar has been widely used in medicine and has many benefits for health, especially vinegar from fruits, such as apple cider vinegar (ACV). ACV contains bioactive components of polyphenols, such as gallic acid, catechin, caffeic acid, and ferulic acid [16, 17]. Research supports ACV has a variety of pharmacological functions, including antioxidant, anti-diabetic, anti-hyperlipidemic, antimicrobial, and anti-inflammatory properties in animal models [18, 19, 20]. A systematic review and meta-analysis of all published clinical trials of ACV consumption significantly decrease total cholesterol, and triglyceride and increase HDL-C concentrations in apparently healthy participants and decreased glucose levels in healthy and a subgroup of patients with Type 2 diabetes [21]. Phenolic compounds are commonly found in the rind of the fruit and can reduce oxidation in the body of the consumer. Mangosteen is an important source of natural phenolic antioxidants which possess biological and medicinal properties [22].

In this study, pressurized hot water, steamed with a pressure of 15 psi for 15 min at a temperature of 121 °C was used to press the phenolic compound from mangosteen rind to fresh to increase the bioactive compounds of mangosteen vinegar. Firstly, total phenolic content, total flavonoid content, and the antioxidant properties of FMR (fresh mangosteen rind), FMF (fresh mangosteen flesh), SMR (steamed mangosteen rind) and SMF (steamed mangosteen flesh) were used to compare for antioxidant properties of mangosteen raw materials prior to mangosteen vinegar processing. Mangosteen rind vinegar (MRV), mangosteen flesh vinegar (MFV), and mangosteen rind plus flesh vinegar (MRFV) were examined. To investigate the quality by assessing the properties of mangosteen vinegar according to the Notification of the Ministry of Public Health, Thailand (No. 204) B.E. 2543 (2000) Re: Vinegar) [23]. Then, we analyzed mangosteen vinegar in terms of total soluble acid, alcohol content, total acid % as acetic acid, and pH for MRV, MFV, and MRFV, and compared it with those of apple cider vinegar (ACV) as the benchmark. The quantitative analysis of MRV, MFV, and MRFV in terms of total phenolic content, total flavonoid content, and antioxidant properties were performed. The phenolic compounds: Gallic acid, Catechin, Epicatechin, Vanillic acid, Tran s-ferulic acid, Rutin, Gamma-mangosteen, and Alpha-mangostin were examined for MRV, MFV, MRFV and ACV using HPLC. We used HPLC to separate, identify and quantify each phenolic compound of the extracts in mangosteen vinegar to compare with ACV which has been reported to enrich phenolic compounds [24]. Finally, the 9-point Hedonic scale was used to assess the sensory test of the mangosteen vinegar compared to ACV.

## 2 Materials and methods

### 2.1 Chemicals and reagents

Analytical grade reagents and chemicals were used in this study except and until cited otherwise. Folin-ciocalteau reagent (Cat No. 1090010500) 2,2-diphenyl-1-picrylhydrazyl (DPPH, Cat No. 1898-66-4), ABTS (2,2′-azino-bis (3-ethylbenzothi-azoline-6-sulfonic acid), diammonium salt, ethanol (90%), gallic acid, potassium persulfate, catechin (Cat No. 154-23-4), epicatechin (Cat No. 490-46-0), vanillic acid (Cat No. 121-34-6), trans-ferulic acid (99%, Cat No. 537-98-4), rutin (Cat No. 250249-75-3), aluminium chloride (AlCl_3_), gamma-mangostin (Cat No. 31271-07-5), alpha-mangostin (Cat No. 6147-11-1), potassium acetate (CH_3_COOK, ACS reagent, ≥99.0%), sodium phosphate (Na_2_CO_3_), and methanol (99.99%) were procured from Sigma-Aldrich (Sigma-Aldrich, Inc. PO Box 14508, St. Louis, MO 68178, United States) through local supplier.

### 2.2 Mangosteen preparation before fermentation

Ripe mangosteen (only purple black, a final ripening stage) fruits harvested from an agroforestry farm in Phrom Khiri, Nakhon Si Thammarat, Thailand, was selected [3]. The No. 01552-4 were Walailak herbarium numbers of mangosteen. Mangosteen. fruits were washed with distilled water and steamed in the autoclave (ALP, Tokyo, Japan), at a pressure of 15 psi for 15 min at a temperature of 121 °C, a pressurized hot water extraction (PHWE), a modification technique of the green process of recovery of bioactive compounds [25]. Then, the steamed mangosteen was divided into 3 types: steamed mangosteen rind (SMR), steamed mangosteen flesh (SMF), and steamed mangosteen rind plus flesh (SMRF; 1:1) to process the mangosteen extract for antioxidant activities test compared to fresh mangosteen extract. The aqueous: ethanol (90:10) solvent was used to shake for fresh mangosteen rind (FMR), fresh mangosteen flesh (FMF), and fresh mangosteen rind plus flesh (FMRF; 1:1) and steamed mangosteen rind (SMR), steamed mangosteen flesh (SMF), and steamed mangosteen rind plus flesh (SMRF; 1:1) for 24 h and filtered with Whatman filter paper No.1 (Sigma-Aldrich, 90mm diameter). The extracted solutions were lyophilized (Ella lyophilizer, Kyoto, Japan). The extracts were stored at −20 °C until further use. The characteristics of steamed mangosteen were observed at 0 h and after standing at room temperature for 3 h and were investigated bacterial growth on enrichment media of nutrient agar to compare before and after steaming of the mangosteen fruit prior to fermentation and vinegar processing.

### 2.3 Vinegar processing of steaming mangosteen

The steamed mangosteen; steamed mangosteen rind (SMR), steamed mangosteen flesh (SMF), and steamed mangosteen rind plus flesh (SMRF; 1:1) were prepared for fermentation processing (mangosteen wine) using the ratio of 1:1:10 of mangosteen: sugarcane: water, respectively. Then, it was fermented with yeast, *Saccharomyces cerevisiae* (TISTR5019, Thailand Institute of Scientific and Technological Research (TISTR) (Cat No 5019) to produce alcohol for 2–3 weeks. The mangosteen wine containing 10–12% alcohol was further incubated with *Acetobacter aceti* (TISTR354, Thailand Institute of Scientific and Technological Research (TISTR) (Cat No 354) for 2–3 weeks to turn alcohol to vinegar with an acetic acid content of at least 4% (w/v) following the Notification of the Ministry of Public Health (No. 204) B.E. 2543 (2000) Re: Vinegar, and Codex Alimentarius Commission (FAO/WHO, 2000) [23,26]. The mangosteen vinegar processing was modified following Saithong et al. [27] as shown in Figure 1.

**Figure 1:** Vinegar processing of steamed mangosteen. MRV, mangosteen rind vinegar; MFV, mangosteen flesh vinegar; MRFV, mangosteen rind plus flesh vinegar.

### 2.4 Determination of mangosteen vinegar qualities

The mangosteen rind vinegar (MRV), mangosteen flesh vinegar (MFV), and mangosteen rind plus flesh vinegar (MRFV) products were taken to measure the quality and physical properties. Total soluble solid (°Brix), alcohol content (%), total acid (%TA) as acetic acid, and pH were analyzed following the guidance of the Association of Official Analytical Chemists (AOAC) (2000) [28]. To determine the color of the mangosteen vinegar, we followed a modified method using a Colorgard System 2000 Colorimeter (BYK-Gardner, Geretsried, Germany), as described by de Beer et al. [29], Where L∗ describes the brightness 0–100 (dark to bright), a∗ describes the color from green (−a∗) to red (+a∗), and b∗ describes the colors from blue (−b∗) to yellow (+b∗). The colorimeter was calibrated before useed with a non-diffusing black reflectance standard (BYKGardner, Geretsried, Germany).

### 2.5 Determination of polyphenols and antioxidant properties

#### 2.5.1 Sample preparation

Mangosteen vinegar, mangosteen rind vinegar (MRV), mangosteen flesh vinegar (MFV), and mangosteen rind plus flesh vinegar (MRFV) were lyophilized (Ella lyophilizer, Kyoto, Japan) for 18 h. The extracts were kept at −20 °*C prior* to use. Apple cider vinegar (ACV), an imported product, was purchased from a supermarket in Nakhon Si Thammarat, Thailand, was lyophilized (Ella lyophilizer, Kyoto, Japan) and was used for comparison. All reagents and chemicals were purchased from Sigma-Aldrich (St. Louis, MO, USA).

#### 2.5.2 Determination of total phenolic content

The total phenolic content of fresh mangosteen, steamed mangosteen, and mangosteen vinegar extracts were determined with the Folin–Ciocalteu reagent using the modified methods [30]. Briefly, 100 μL Folin–Ciocalteu reagent was mixed with 20 μL of mangosteen sample or the standard set of gallic acid and incubated at room temperature for 5 min. Then, 300 μL Na_2_CO_3_ (25%w/v) was mixed and incubated at 45 °C for 30 min. The absorbance of the sample and standard were measured at a wavelength of 765 nm using a UV-visible spectrophotometer (V-630, JASCO, Tokyo, Japan). Results were expressed as milligram of gallic acid equivalent per gram dry weight (mgGAE/g extracted). All the determination tests were carried out in triplicate.

#### 2.5.3 Determination of total flavonoid content

The aluminum chloride colorimetric method was used for the determination of the total flavonoid content of the samples following the modified method of Chowdhury et al. [31]. Briefly, mangosteen extracts or standard solutions of quercetin were prepared by serial dilutions using methanol mixed with 3 mL of methanol (99.99%), 0.2 mL of 10% AlCl_3_ (w/v), 0.2 mL of 1 M potassium acetate (CH_3_COOK), and 5.6 mL of distilled water and then incubated at room temperature for 30 min. The absorbance of the reaction mixture was measured at 415 nm with a UV-visible spectrophotometer (UV-1280, Shimadzu, Kyoto Japan) against a methanol blank. The flavonoid content was calculated and expressed in milligram quercetin per gram dry weight (mgQE/g extracted). All the determination tests were carried out in triplicate.

#### 2.5.4 Antioxidant properties by DPPH assay

Testing for antioxidant activity by 2,2-diphenyl-1-picrylhydrazyl (DPPH) radical scavenging activity was performed with modifications according to Hiransai et al. [32]. Briefly, we added 100 μL of different concentrations of mangosteen vinegar with 200 μL of methanolic solution of DPPH 0.1 mM into a 96-well microplate in triplicates. The mixture was incubated for 60 min at room temperature and protected from light. The DPPH scavenging activity of mangosteen vinegar was measured at 517 nm by a microplate reader (EON, BioTek, Vermont, USA) against a blank. The antioxidants in extracts were calculated as the inhibitory concentration (IC50, μg/mL).

#### 2.5.5 Antioxidant properties by ABTS assay

Testing for antioxidant activity by 2,2′-azino-bis (3-ethylbenzthiazoline-6-sulphonic acid) (ABTS) radical cation decolorization assay used the modified method of Re et al. [33]. Briefly, 7 mM ABTS was placed in H_2_O with 2.45 mM potassiumpersulfate (K_2_S_2_O_8_) and incubated for 18 h. The resulting ABTS radical solution was diluted in distilled water, and the optical density was determined at 415 nm with a UV-visible spectrophotometer (UV-1280, Shimadzu, Kyoto Japan). Then, 180 μL of ABTS + solution was reacted with 20 μL of different concentrations of mangosteen vinegar for 15 min at room temperature and protected from light. The absorbance of the reaction mixture was determined at 415 nm and was calculated the antagonist 50% inhibitory concentration (IC50, μg/mL).

#### 2.5.6 Determination of the phenolic compounds using HPLC

MRV, MFV, MRFV, and ACV extracts were soaked in 50% methanol. The phenolic compounds of the extracts were determined quantitatively by the reverse phase HPLC system (Prominence-I LC-2030C 3D Plus, Shimadzu, Kyoto, Japan) coupled with a Shim-pack GIST C-18 column (4.6 × 150 mm, 5 μm size (Shimadzu Corporation, Tokyo, Japan)), and a photodiode array detector (SPD-M30A, Shimadzu Corporation, Japan) was used to identify the phenolic contents of the extracts [34, 35]. The C-18 column was used as a stationary phase while the mobile phase consisted of elution gradient 2% acetic acid in water and methanol (HPLC grade >99.9%; Sigma-Aldrich Co. St Louis, USA), with a flow rate of 1.0 mL/min. A volume of 20 μL was injected. Compounds separation was monitored at a wavelength of 278 nm. All the identified peaks in this work were eluted within 60 min. Catechin, epicatechin, vanillic acid, trans-ferulic acid, rutin, gamma-mangostin, and alpha-mangostin were used as the standard phenolic compounds evaluated in this study. ACV was used as a benchmark.

### 2.6 Sensory evaluation

For the sensory evaluation of the mangosteen vinegar, MRV, MFV, and MRFV were prepared in 50% concentrations in drinking water. The sensory panel members (n = 30, age 36.4 ± 8.5 years), based on the 9-point Hedonic scale, were trained to distinguish, and evaluate all aspects of taste, flavor, and texture of food products. The apple cider vinegar (APC) was used as a benchmark. Samples were evaluated by the panel members in terms of appearance, such as cloudiness properties, color, aroma, taste, texture, and overall acceptability by using the 9-point Hedonic scorecard for each vinegar [36]. The sensory evaluation test of the mangosteen vinegar was approved by the Walailak University Human Ethics Approval Committee (WUEC-21-254-01) and was tested on 30 volunteers. The informed consent was obtained from the participants before sensory evaluation experiments.

### 2.7 Statistical analysis

Data are presented as mean ± standard error of mean (SEM) of three independent experiments. One-way ANOVA was used for analysis and followed by Tukey's multiple comparison post hoc test (GraphPad Prism 4, San Diego, CA. USA). A *p* < 0.05 is statistically significant.

## 3 Results and discussion

### 3.1 Mangosteen preparation before fermentation

Washed mangosteen fruits were blanched by steaming in the autoclave at a pressure of 15 psi for 15 min at a temperature of 121 °C. The characteristics of fresh and steamed mangosteen were observed at 0 h and 3 h, and the results are shown in Figure 2A–D. It is well known that the browning of fresh fruit and vegetables reduces the quality of products [37]. The fresh mangosteen 3 h after peeling changed in appearance to brown, as shown in Figure 2A, B. It has been reported that polyphenol oxidase (PPO) and peroxidase (POD) can reduce the polyphenolic content in fruits and vegetables by 90% from the initial level [37, 38, 39]. Heat has been shown in the inactivation of PPO and POD as a function of water activity and requires more than 15 min at 80 °C for 50% loss of activity [40, 41]. The purpose of steaming the mangosteen under pressurized hot water extraction (PHWE) was to replace traditional steam distillation and to inhibit enzyme activity. Steaming can reduce degradation from enzymatic causes such as the browning reaction and rancidity from hydrolytic rancidity [25, 42]. Therefore, the present study found that the appearance of streamed mangosteen after peeling for 3 h was not changed compared with at 0 h as Figure 2C, D. In the process of preparing raw material for fermentation of mangosteen using high-pressure hot water, which can inhibit the enzyme activity, the color remained a bright purple. This innovative processing can transfer a purple color from the rind to the flesh (Figure 2C, D).

**Figure 2:** The stability of fresh mangosteen and streamed mangosteen after peeling (A) fresh mangosteen (0 h); (B) fresh mangosteen (3 h); (C) steamed mangosteen (0 h); (D) steamed mangosteen (3 h).

Moreover, high-pressure hot water (HHPW) steaming of mangosteen can inhibit the bacteria growth, as shown in Figure 3R1 and F1 compared to R2 and F2, respectively before and after streamed mangosteen rind and fresh. Our results confirmed that steamed mangosteen using the autoclave at a pressure of 15 psi for 15 min at the temperature of 121 °C in order to remove the contaminated bacteria, inhibited the enzyme polyphenol oxidase activity and facilitated the moving of phenolic contents from mangosteen rind to flesh.

**Figure 3:** Bacterial culture of mangosteen before and after steaming: R1 and R2 are before and after steaming of mangosteen rind; F1 and F2 are before and after steaming of mangosteen flesh.

### 3.2 Total phenolic content, total flavonoid content, and antioxidant properties of fresh and steamed mangosteen

The antioxidants of the FMR, SMR, FMF, and SMF were analyzed (Table 1). The data of the total phenolic content, total flavonoid content, and the antioxidant capacity was reported using ABTS and DPPH scavenging assays found in the mangosteen before vinegar fermentation. Total phenolic content, flavonoid content, and antioxidant activity showed the highest in order of MRV > MRVF > MVF > ACV, respectively. Applications of pressurized hot water using the autoclave at a temperature of 121 °C for 15 psi and a short time of 15 min increased the amount of the phenolic content from mangosteen rind moved to the flesh. Table 1 shows significantly increased total phenolic content, total flavonoid content, and antioxidant activity in the steamed mangosteen flesh (FMR) compared with the fresh mangosteen flesh (FMF) (*p* < 0.05). It was evident that the extraction of SMF by applying heat and pressure increased the amount of phenolic content higher than in FMF. This was consistent with studies of Zhang et al. [43] which applied pressure and found that heat high hydrostatic pressure assisted extraction was revealed to be the suitable technique for phenolic extraction compared to other methods such as ultrasonic-assisted extraction (UE) and microwave-assisted extraction (ME). Thus, the increased rise in pressure and heat quickly transferred the important substances such as total phenolic content and total flavonoid content from the rind to the flesh (Table 1).

**Table 1:** Total phenolic content, total flavonoid content, and antioxidant properties of fresh and steamed mangosteen extract.

Mangosteen extracts	Total phenolic content (mgGAE/g extracted)	Total flavonoid content (mgQE/g extracted)	IC_50_ (μg/mL)	
			ABTS	DPPH
FMR	1208.22 ± 4.90	2.8 ± 0.01	5.54 ± 0.01^c^	1.80 ± 0.01^c^
FMF	225.78 ± 3.29	0.05 ± 0.01	140.39 ± 0.06^c^	82.52 ± 0.06^c^
SMR	945.44 ± 6.90^a^	1.44 ± 0.01^a^	10.86 ± 0.02^a^^,^^c^	2.94 ± 0.09^c^
SMF	359.78 ± 4.00^b^	0.19 ± 0.01^b^	24.26 ± 0.01^b^^,^^c^	12.68 ± 0.02^b^^,^^c^
Ascorbic acid	–	–	0.21 ± 0.01	42.16 ± 0.03

Data are presented as mean ± SEM of three independent experiments.

a *p* < 0.05, compared between fresh and steamed mangosteen rind extract.

b *p* < 0.05, compared between fresh and steamed mangosteen flesh extract.

c *p* < 0.05, compared between fresh and steamed mangosteen extracts and ascorbic acid. FMR, fresh mangosteen rind; FMF, fresh mangosteen flesh; SMR, steamed mangosteen rind; SMF; steamed mangosteen flesh.

The antioxidant activity was determined in terms of IC50 of the free radical scavenging assay (2, 2′-azino-bis-3-ethylbenzthiazoline-6-sulphonic acid) (ABTS) radical cation decolorization assay, and the ability in the binding of free radicals (2,2-diphenyl-1-picrylhydrazyl (DPPH) radical scavenging activity) (Table 1). The results showed that FMR presents the highest ability of ABTS antioxidant activity and capacity to achieve binding of free radicals of DPPH higher than ascorbic acid (*p* < 0. 05). However, we found that the total phenolic content, total flavonoid content, and antioxidant activity of the SMF were higher than FMF after steaming according to applying heat and pressure. This finding will be a benefit for the development of mangosteen flesh products including vinegar.

### 3.3 Qualities of mangosteen vinegar

Table 2 shows the total soluble solid (°Brix) of MFV and MRFV significantly higher than in MRV and ACV indicating that the concentration of sugar in MFV and MRFV is higher than in MRV and ACV (*p* < 0. 05). These soluble solids in fruits are primarily sugars; sucrose, fructose, and glucose which mangosteen flesh contains sugar, 16 g/100 g food value per 100 g of edible portion, more than the peel [44]. The first step of alcoholic fermentation by *Saccharomyces cerevisiae* (TISTR5019) produced mangosteen wine. The second stage of fermentation by *Acetobacter aceti* (TISTR354) completely changed the alcohol to acid and reached the Ministry of Public Health (MOHP) of Thailand No. 204 BE 2543 (2000) [23] standard requirement of % of acetic acid of vinegar (>4%), as in Table 2. The pH of the mangosteen vinegar in the second stage of fermentation of *A. aceti* will notice an increase in acidity in MRV, MFV, and MRFV showed significantly lower than ACV (*p* < 0. 05). Thus, lowering the pH due to the accumulation of acetic acid and organic acids such as tartaric, propionic acid, and vanillic acid which is vital for the development of the flavor and aroma of vinegar [45]. To test the stability of pH and found that the pH in the mangosteen vinegar was not changed after 15 days (data not shown) as the standard of the quality of fruit vinegars specified by the Ministry of Public Health of Thailand, No. 204 (2000) and pH ranged from 2.40 to 3.90, the same values had been reported by the other of fruits vinegar [46, 47]. Color is derived from the natural pigments in fruits which change as the plant proceeds through maturation and ripening [48]. The color of vinegar is a parameter of the quality of natural vinegar. Mangosteen vinegar showed brightness (L∗) and a red-yellow color stronger than ACV, as in Table 2. It is well known that mangosteen ripening peel contains the water-soluble anthocyanins (red) and flavonoids (yellow) [7]. In addition, the processing of vinegar step of preparation raw mangosteen material using autoclave, high hot pressure, inhibited the enzymes involved in browning reactions including polyphenol oxidase which catalyzes the oxidation of polyphenolic compounds [40, 41]. Mangosteen vinegars that have been shown weakness in red (+a∗) and strongest yellow (+b∗) indicating that anthocyanins are sensitive to both pH and heat, while the flavonoids are sensitive to oxidation by PPO and POD enzymatic reactions which were inhibited by high hot-pressure steaming process in the preparation of the raw materials. This study is consistent with the previous study which showed the effects of vinegar extraction from mangosteen peel in the same manner [49].

**Table 2:** The qualitative analysis results of MRV, MFV, MRFV, and ACV.

Parameters		Treatments			
		MRV	MFV	MRFV	ACV
Total soluble solid (°Brix)		1.30 ± 0.00	4.20 ± 0.00^a^^,^^b^	5.00 ± 0.00^a^^,^^b^	1.10 ± 0.00
Alcohol content (%)		0.00	0.00	0.00	0.00
Total acid (%TA) as acetic acid		5.01 ± 0.74	4.96 ± 0.89	4.91 ± 0.36	5.00 ± 0.00
pH		2.27 ± 0.00^a^	3.10 ± 0.00^a^^,^^b^	2.17 ± 0.00^a^	4.16 ± 0.00
Color	L∗	5.17 ± 0.12^a^	2.60 ± 0.04^a^^,^^b^	2.10 ± 0.06^a^^,^^b^	1.10 ± 0.09
	a∗	1.44 ± 0.39^a^	1.29 ± 0.21^a^^,^^b^	0.52 ± 0.34^a^^,^^b^	0.02 ± 0.18
	b∗	7.77 ± 0.35^a^	2.65 ± 0.33^a^^,^^b^	3.65 ± 0.57^a^^,^^b^	0.96 ± 0.45

Data are presented as mean ± SEM of three independent experiments.

a *p* < 0.05 comparing mangosteen vinegar to ACV.

b *p* < 0.05 indicates significant differences within the mangosteen vinegar group. MRV, mangosteen rind vinegar; MFV, mangosteen flesh vinegar; MRFV, mangosteen rind plus flesh vinegar; ACV, apple cider vinegar. L∗, brightness 0–100 (dark to bright); a∗, red (+a∗) to green (−a∗); b∗, yellow (+b∗) to blue (−b∗).

### 3.4 The phenolic compound and antioxidant properties of vinegar fermentation

Table 3 shows the total phenolic and total flavonoid contents in the extracts of mangosteen flesh vinegar (MFV), mangosteen rind vinegar (MRV), and mangosteen flesh plus rind vinegar (MFRV) showed significantly higher levels than apple cider vinegar (ACV) (*p* < 0. 05). These results correlate to the antioxidant activity of MRV, MFV, and MRFV in the potent scavenging of free radicals ABTS+ and DPPH. Moreover, MRV, MFV, and MRFV showed higher scavenging of free radicals of ABTS+ and DPPH- than ACV and ascorbic acid (*p* < 0.05) as Table 3. It is anticipated that the phenolic compound is relatively stable and constitutes competition to reduce the number of free radicals [50]. Applications of pressurized hot water extraction (PHWE) for the extraction of bioactive compounds such as phenolic compounds from fruits and plants using water temperatures of 80–175 °C and short extraction times have been reported to increase higher antioxidant capacity [51, 52, 53]. Taken together, suggested that MVR, MVF, and MRFV processed under the condition of high-pressure hot water remained the higher antioxidant activity.

**Table 3:** Total phenolic content, total flavonoid content, and antioxidant properties of MRV, MFV, MRFV, and ACV.

Extracts	Total phenolic content (mg GAE/g extracted)	Total flavonoid content (mg QE/g extracte)	IC50 (μg/mL/	
			ABTS	DPPH
MRV	175.69 ± 19.60^a^	0.26 ± 0.01^a^	84.93 ± 0.04^a^^,^	12.74 ± 0.02^a^^,^^b^^,^^c^
MFV	541.40 ± 18.80^a^^,^^b^	0.21 ± 0.01^a^	101.21 ± 0.01^a^^,^^b^	40.19 ± 0.06^a^^,^^b^
MRFV	702.30 ± 5.80^a^^,^^b^	0.25 ± 0.01^a^	95.22 ± 0.42^a^^,^^b^	15.76 ± 0.06^a^^,^^b^^,^^c^
ACV	460.36 ± 3.90	0.12 ± 0.01	110.48 ± 0.12	93.71 ± 0.06^c^
Ascorbic acid		–	0.21 ± 0.01	42.16 ± 0.31

Data are presented as mean ± SEM of three independent experiments.

a *p* < 0.05 compared with ACV.

b *p* < 0.05 compared within the mangosteen vinegar group.

c *p* < 0.05 compared with ascorbic acid. MRV, mangosteen rind vinegar; MFV, mangosteen flesh vinegar; MRFV, mangosteen rind plus flesh vinegar; ACV, apple cider vinegar.

### 3.5 Determination of phenolic compounds by high-performance liquid chromatography (HPLC)

HPLC, a conventional method, was used to separate and identify the phenolic compounds in mangosteen vinegar and apple cider vinegar as shown in Table 4. Table 4 shows that gallic acid, epicatechin, vanillic acid, trans-ferulic acid, and rutin were detected in relatively high concentrations in MRV, MFV, and MRFV, significantly higher than found in ACV (*p* < 0. 05). The phenolic compound found in lower concentrations compared to ACV (*p* < 0.05) was catechin. Plaza et al. found that the highest yield of quercetin extraction is at 175 °C, 5 min extraction time, and it is not very soluble in water at room temperature [51] which may be the same as in us extraction conditions (121 °C, 15 psi, 15 min). Importantly xanthone derivative, gamma-mangostin was found the highest level in MFV compared to MRV, MRFV and ACV (*p* < 0. 05). Moreover, Gamma-mangostin showed a potent antioxidant free radical scavenging significantly higher than in ACV (*p* < 0. 05). Application of high-pressure hot water supported our aim to transfer phenolic compounds from rind to flesh, especially gamma-mangostin, as shown in Table 4. Vanillic acid extract was detected in mangosteen vinegar in significantly higher amounts than found in ACV. Vanillic acid affects the production of vinegar in terms of smell, and vinegar made from mangosteen has a very strong fruit smell [54]. Vanillic acid has been suggested to have the ability to inhibit inflammation and fight cancer by reducing the number of cancer cells in the small intestine [55, 56]. It is well-known that functional foods have an impact on human health [57]. MFV showed potent scavenging of free radicals and antioxidants that should be further studied regarding their effects on inflammation and chronic diseases such as cancer, diabetes, and cardiovascular and neurodegenerative diseases.

**Table 4:** Phenolic compounds of MRV, MFV, MRFV, and ACV determined using HPLC.

Extracts phenolic compound (mg/kg)	MRV	MFV	MRFV	ACV
Gallic acid	84.72 ± 14.02^a^	243.84 ± 13.04^a^^,^^b^	55.04 ± 5.04^a^	35.98 ± 3.50
Catechin	446.46 ± 26.46^a^	342.17 ± 23.27^a^^,^^b^	345.92 ± 25.09^a^^,^^b^	810.04 ± 18.01
Epicatechin	937.69 ± 9.37^a^	2049.95 ± 20.49^a^^,^^b^	1010.29 ± 30.10^a^^,^^b^	842.43 ± 18.42
Vanillic acid	2487.98 ± 24.56^a^	2653.60 ± 26.35^a^^,^^b^	1912.43 ± 21.91^a^^,^^b^	199.36 ± 9.99
Trans-ferulic acid	18359.47 ± 38.95^a^	2134.10 ± 21.43^a^^,^^b^	9348.09 ± 29.94^a^^,^^b^	109.89 ± 9.80
Rutin	13266.51 ± 153.32^a^	5976.30 ± 49.67^a^^,^^b^	5257.16 ± 52.61^a^^,^^b^	206.04 ± 16.08
Gamma-mangostin	29.95 ± 2.69	373.20 ± 3.65^a^^,^^b^	37.77 ± 4.78	38.00 ± 4.68
Alpha-mangostin	19.00 ± 0.85^a^	LoD	8.10 ± 0.54^a^	LoD

Data are presented as mean ± SEM of three independent experiments.

a *p* < 0.05 indicates significant differences compared with ACV.

b *p* < 0.05 indicates significant differences among mangosteen vinegars. LoD; Lower limit of detection.

### 3.6 Sensory evaluation

The results of the sensory evaluation of the vinegars and a blend of the vinegars and water (1:1), based on the 9- point Hedonic scale, are depicted in Table 5. Appearance and color, derived from the natural pigments in ripening mangosteen, were preserved in MVR, MFV, and MRFV, significantly more than in ACV (Table 5). Significant differences in color were observed among the mangosteen vinegar products and MFV displayed the highest level of panelists' preference in terms of color (7.13 ± 1.43). The application of high temperature and pressure of 121 °C and 15 psi, for 15 min to steam ripe mangosteen transferred color from the rind to flesh and inhibited PPO and POD enzyme activities by stopping browning reactions, as shown in Figures 1 and 2. Moreover, the MFV displayed the highest level of panelists' preference, with a mean overall acceptability score of 6.73 ± 1.82 (Table 5). The other parameters including aroma, test, texture, and overall acceptability were the highest on the scale (Table 5). The 9-point Hedonic scale has been the primary method of scaling in food sensory evaluation and has been widely used for the assessment of consumers’ acceptability of foods and drinks [58]. Color and appearance attract the consumer to a product and aroma, test, texture, and flavor quality influence impulse purchases [59].

**Table 5:** Sensory evaluation of MRV, MFV, MRFV, and ACV using the 9-point Hedonic scale.

Parameters	MRV	MFV	MRFV	ACV
Appearance	7.17 ± 0.25^a^	6.97 ± 0.22^a^	7.23 ± 0.21^a^	6.50 ± 0.31
Color	6.53 ± 0.38	7.13 ± 0.26^a^^,^^b^	7.00 ± 0.26^a^^,^^b^	6.63 ± 0.26
Aroma	6.10 ± 0.32^a^	6.17 ± 0.32^a^	5.77 ± 0.34^b^	5.30 ± 0.43
Taste	5.47 ± 0.44	5.83 ± 0.39^a^,^b^	5.80 ± 0.44^a^^,^^b^	5.13 ± 0.43
Texture	6.07 ± 0.39	6.40 ± 0.33^a^^,^^b^	6.17 ± 0.38	5.87 ± 0.41
Overall acceptability	6.03 ± 0.46^a^	6.73 ± 0.33^a^^,^^b^	6.00 ± 0.38^a^	5.47 ± 0.36^c^

Data are presented as mean ± SEM of three independent experiments.

a *p* < 0.05 indicates significant differences compared with ACV.

b *p* < 0.05 indicates significant differences among mangosteen vinegars.

## 4 Conclusions

This study demonstrated the development of a method for processing mangosteen vinegar from ripe-black colored mangosteen containing the highest total phenolic contents. An application to steam mangosteen under pressurized hot water extraction (PHWE) was developed to increase the content of phenolic compounds from the mangosteen peel into the mangosteen flesh using the extraction process through high heat and pressure. This process enhanced the vinegar's antioxidant ability, and the level of consumer acceptability for mangosteen vinegars proved to be higher than apple cider vinegar. Based on the scavenging effect, the chronology of antioxidant capacity of the vinegar is found to be MRV > MRFV > MFV > ACV. Furthermore, this work provides a new approach to processing ripe mangosteen byproducts that contributes to the value-added products and the high-quality beneficial effects of mangosteen vinegar.

## Declarations

### Author contribution statement

Nathamon Suksamran; Visaka Anantawat; Jitbanjong Tangpong: Conceived and designed the experiments; Performed the experiments; Analyzed and interpreted the data; Contributed reagents, materials, analysis tools or data; Wrote the paper.

Phanphen Wattanaarsakit; Hideyuki J. Majima: Contributed reagents, materials, analysis tools or data; Wrote the paper.

Chen Wei; Md. Atiar Rahman: Analyzed and interpreted the data; Contributed reagents, materials, analysis tools or data; Wrote the paper.

### Funding statement

This work was supported by 10.13039/501100010034Walailak University, Thailand scholarship on contract no. 05/2559 and no. 21/2562.

### Data availability statement

Data will be made available on request.

### Declaration of interest's statement

The authors declare no conflict of interest.

### Additional information

No additional information is available for this paper.
